The article "Metabolic Syndrome: Lessons from Rodent and Drosophila Models" was published in 2022. Journal: Biomed Res Int.

# Metabolic Syndrome: Lessons from Rodent and *Drosophila* Models

**DOI:** 10.1155/2022/5850507

**Published:** 2022-06-22

**Authors:** Myroslava V. Vatashchuk, Maria M. Bayliak, Viktoria V. Hurza, Kenneth B. Storey, Volodymyr I. Lushchak

**Affiliations:** ^1^Department of Biochemistry and Biotechnology, Vasyl Stefanyk Precarpathian National University, 57 Shevchenko Str., Ivano-Frankivsk 76018, Ukraine; ^2^Institute of Biochemistry, Carleton University, 1125 Colonel By Drive, Ottawa, Ontario, Canada K1S 5B6; ^3^Research and Development University, Shota Rustaveli Str., 76018 Ivano-Frankivsk, Ukraine

## Abstract

Overweight and obesity are health conditions tightly related to a number of metabolic complications collectively called “metabolic syndrome” (MetS). Clinical diagnosis of MetS includes the presence of the increased waist circumference or so-called abdominal obesity, reduced high density lipoprotein level, elevated blood pressure, and increased blood glucose and triacylglyceride levels. Different approaches, including diet-induced and genetically induced animal models, have been developed to study MetS pathogenesis and underlying mechanisms. Studies of metabolic disturbances in the fruit fly *Drosophila* and mammalian models along with humans have demonstrated that fruit flies and small mammalian models like rats and mice have many similarities with humans in basic metabolic functions and share many molecular mechanisms which regulate these metabolic processes. In this paper, we describe diet-induced, chemically and genetically induced animal models of the MetS. The advantages and limitations of rodent and *Drosophila* models of MetS and obesity are also analyzed.

## 1. Concept of Metabolic Syndrome

Metabolic syndrome (MetS) is a combination of metabolic abnormalities that increases the risk of cardiovascular diseases, diabetes, stroke, and other pathologies. These abnormalities include central obesity, hypertension, insulin resistance, and atherogenic dyslipidemia [1]. Approximately 20–30% of the adult population in most countries is estimated to suffer from MetS. The prevalence depends on age, gender, race, and diagnostic criteria. The incidence of MetS is expected to increase to approximately 53% by 2035 [2].

The clustering of several metabolic abnormalities within an individual was first discussed by Dr. Reaven in 1988. This clinical phenotype has been given different names over the years such as “insulin resistance syndrome,” “syndrome X,” “hypertriglyceridemic waist,” and “the deadly quartet.” But now, it is most commonly called “metabolic syndrome” [3] and is increasingly recognized as an important cardiovascular risk factor [1].

In 1999, the WHO published the definition of metabolic syndrome based on the assumption that development of insulin resistance and impaired glucose regulation is among the major factors contributed to MetS. The definition states that to diagnose a patient with MetS, the presence of two additional risk factors should be confirmed from a list that includes hypertension, central obesity, increased levels of blood triacylglycerides (TAG), or low levels of high density lipoproteins (HDL) [4]. Over the last few decades, the leading world health organizations such as the European Group on Insulin Resistance (EGIR), the International Diabetes Federation (IDF), the American Association of Clinical Endocrinologists (AACE), the American Heart Association (AHA), and the National Heart, Lung, and Blood Institute (NHLBI) improved the definition of MetS and changed its criteria [4–6]. In 2009, IDF, NHBLI, AHA, WHO, and the International Association for the Study of Obesity published a joint definition of MetS. The definition states that “to diagnose with the MetS the presence of 3 out of 5 signs is required: increased waist circumference, taking into account specific criteria for the population and individual countries, elevated levels of blood TAGs, low levels of HDL, high blood pressure, and hyperglycemia” [6].

As a multifactorial condition with an endangered rate of spread, MetS requires the development of appropriate experimental models in animals that mimic the disease state to address the difficulty of assessing the pathophysiology of MetS in humans. Rats and mice are the most common models used in the study of MetS [7, 8]. In recent years, the fruit fly, *Drosophila melanogaster*, has become an emerging model to explore metabolic disturbances and obesity-related disorders in a cost-effective and expedient manner [9, 10]. In this review, we discuss various rodent and fly models of MetS highlighting their advantages and limitations. Generally, studies of obesity and MetS in *Drosophila* and rodent models have shown that flies and small mammal models have many similarities with humans in basic metabolic functions and share many molecular mechanisms regulating these metabolic processes. Here, we also provide information on feasibility of using *Drosophila* not only for studying mechanisms underlying MetS but also for testing preventive strategies against obesity and MetS.

## 2. Animal Models in Metabolic Syndrome Research

Different approaches have been developed to study MetS pathogenesis and underlying mechanisms including diet-induced and genetic models of MetS (Table 1 and Figure 1).

### 2.1. Diet-Induced Models

Feeding with high caloric food rich in fats or carbohydrates or both is a popular and effective approach to induce metabolic abnormalities in laboratory animals [8].

#### 2.1.1. Rodents

It is not surprising that mammalian models are widely used to study different aspects of MetS since they share many functional and metabolic similarities with humans. Diet-induced obesity rodent models are most popular for studies of human obesity and related complications such as MetS. To induce the obesity phenotype, animals are fed with different types of high caloric diets, the high-fat diet (typically 40%–60% fat composition) being the most popular. The development of clinical parameters as observed in human MetS patients such as abnormal lipid concentration in plasma coupled with high blood pressure and insulin resistance has been demonstrated in numerous high-fat diet (HFD) studies with rodents [11–16]. In particular, Avtanski et al. [15] found that 9 weeks of HFD intervention, providing 60% energy from fat, resulted in a chronic proinflammatory state and insulin resistance in male C57BL/6J mice. The study of Rahmouni et al. [12] found that C57BL/6J mice on HFD (45% fat) showed higher baseline systolic, diastolic, and mean arterial pressure than the mice on the normal diet (13% fat). Lackey et al. [17] showed that overfeeding a low-fat diet (8.6% energy from fat) resulted in levels of obesity similar to high-fat diet (40.1% energy from fat) feeding in C57BL/6 mice. However, despite a similar body weight, obese HFD mice were more insulin resistant than mice fed with an isocaloric low-fat diet [17]. Feeding Sprague-Dawley rats with HFD (47% calories from fat) increased plasma levels of total cholesterol, triacylglycerides (TAG), and low density lipoproteins (LDL) and decreased high density lipoprotein (HDL) levels as compared with those parameters in rats fed with the control diet (13% calories from fat) [14]. In addition, mice fed with HFD (60%) exhibited significantly increased body mass, total fat pads, plasma TAG, HDL, and LDL cholesterol levels as compared with the control group [7]. A study of the chronic effects of HFD with different fat content (10, 32, and 45%) on body adiposity and metabolism in rats demonstrated that energy intake, weight gain, fat mass, levels of plasma glucose, cholesterol, TAG, free fatty acids, leptin, and insulin increased with increasing content of dietary fat in a dose-dependent manner [18].

Metabolic abnormalities associated with MetS were also registered in studies where rats and mice were fed with high fructose or sucrose diets [7, 19, 20]. In particular, consumption of 10% fructose in drinking water resulted in the same effects as a high dose fructose food diet (60%), and these effects included hypertension and hyperlipidemia in male Sprague-Dawley rats [20]. In C57BL/6 mice, a high-fructose diet (34% fructose) caused multiple symptoms of MetS, such as insulin resistance, impaired glucose tolerance, hyperinsulinemia, hypertension, and hypertriglyceridemia [21]. The study of Cao et al. [22] showed that a diet containing 35% of caloric intake from sucrose led to insulin resistance in Sprague-Dawley rats compared to the control group, whereas body weight did not increase during feeding for 20 weeks. Increasing evidence indicates that high fructose diet causes various features of MetS such as obesity, adiposity, hypertension, hypertriglyceridemia, dyslipidemia, glucose intolerance, and decreased insulin sensitivity [23–25]. Many studies report that fructose is involved more extensively than glucose in nonenzymatic processes and generation of reactive species [26, 27]. Long-term fructose intake has been demonstrated to cause carbonyl/oxidative stress [26, 28] that can contribute to development of MetS complications [29]. Sucrose, glucose, or starch-based feeding was not as effective as feeding with fructose to induce MetS [24, 30]. Mice fed with fructose gained more weight and developed severe MetS signs compared to those fed with the same calories of starch [7, 31]. Thus, it seems that there are some differences between fructose and glucose metabolism, perhaps because these monosaccharides require different enzymes in the initial steps of metabolism [32]. However, it should be noted that a more pronounced impact of glucose over fructose occurred when the sugar was combined with a high-fat diet to induce metabolic changes associated with MetS [33]. Rats fed a high-fat/high-carbohydrate diet demonstrated a greater increase in body weight, fat deposition, oxidative stress biomarkers, fasting levels of blood glucose and insulin, and allodynia (a feature of neuropathic pain) than the control group, suggesting development of MetS in the experimental diet group. These alterations were more pronounced in glucose-fed animals as compared with fructose-fed ones, suggesting a main contribution of glucose to MetS development [33].

Many other studies support the high impact of fructose consumption in MetS development. In rats, the consumption of fructose in drinking water for 12 weeks induced the classic symptoms of the MetS. Rats given the high fructose diet showed a greater significant increase in body mass and had significantly higher levels of blood glucose, serum insulin, total cholesterol, and TAG, as well as higher systolic blood pressure, diastolic blood pressure, and mean arterial pressure compared to the control group that did not receive fructose [34]. In addition, fructose administration increased HOMA-IR index suggesting induction of insulin resistance [34]. A study by Oron-Herman et al. [35] showed that a fructose-enriched diet caused Sprague-Dawley rats (SDRs) to become hyperinsulinemic, hypertriglyceridemic, hypercholesterolemic, hypertensive, and insulin resistant, whereas spontaneously hypertensive rats (SHRs) responded to sucrose supplementation by a significant elevation in blood pressure and mild worsening of insulin resistance.

In male Wistar rats, the consumption of 30% sucrose in drinking water resulted in the development of MetS symptoms such as increased body weight, elevated blood pressure, and increased blood levels of insulin, TAG, total cholesterol, and low-density lipoproteins [36]. Similar results were obtained by Pang et al. [37]; supplementation with 77% sucrose significantly increased systolic blood pressure, plasma insulin, and TAG levels in rats.

Cheng et al. [38] demonstrated that the interplay between the developmental stage of the rats and the type of diet plays a crucial role in disease induction. Three-week old postweaning rats given HFD for eight weeks developed all the phenotypes of MetS whereas adult rats on high-fat-high-sucrose diet (HFSD) merely became obese and hypertensive, making the former a more time-saving and cost-effective MetS model [38].

A modified high-carbohydrate high-fat (HCHF) diet containing 17.5% fructose, 39.5% sweetened condensed milk, 20% ghee, and 15.5% powdered rat food, as well as drinking water supplemented with 25% fructose, led to partial development of components of MetS after 8 weeks of feeding in Wistar rats and fully developed MetS after 12 weeks [20]. The HFD also induced metabolic alterations in C57BL/6 mice similar to those observed in humans with MetS as well as development of nonalcoholic fatty liver disease associated with HFD that is another risk factor for MetS [39]. Increasing age is also an important contributing factor for augmenting such metabolic alterations, mainly obesity and hepatic fat deposition [39].

#### 2.1.2. Drosophila melanogaster

In recent years, the fruit fly *Drosophila melanogaster* has been used as a model for elucidating the mechanisms that regulate fat metabolism, distribution, and deposition. Obese flies accumulate triacylglycerols mainly in the fat body, an organ similar to mammalian adipose tissue, which specializes in lipid storage and catabolism. Furthermore, obese flies exhibit pathophysiological complications, including hyperglycemia, reduced longevity, and cardiovascular function, similar to those observed in obese humans [9, 10, 40]. Insulin-like peptides and adipokinetic hormone (AKH) are two key regulators of carbohydrate and lipid homeostasis in flies. They are analogs of human insulin and glucagon, respectively [10, 41]. *Drosophila* insulin signaling, despite having eight insulin-like peptides with partially redundant functions, is very similar to the human insulin pathway and has served as a model to study many different aspects of diabetes and the diabetic state [42, 43]. One of the advantages of having viable *Drosophila* mutant combinations affecting different levels of the insulin pathway is that the abnormal metabolic state can be studied from the onset of the life cycle and followed throughout [44, 45].

In *D*. *melanogaster*, high carbohydrate diets based on sucrose, glucose, or fructose delayed pupation, increased larval mortality, shortened lifespan, and induced an obese-like phenotype in adults [40, 46, 47]. The latter was characterized by increased fly body mass, higher levels of body triacylglycerols and storage carbohydrates (trehalose, glycogen), and consequences including hyperglycemia, insulin resistance, and increased levels of circulating insulin-like peptides in hemolymph [46–49]. A high-fat diet also caused an obese-like phenotype in adult flies including increased circulating glucose levels and body triacylglycerol content, increased insulin-like peptide resistance, enhanced rates of lipid peroxidation and cardiac lipid accumulation, and reduced cardiac contractility [50–53]. As in mammals, dibutyl phthalate may induce an obese-like phenotype in *Drosophila* that disrupts evolutionarily conserved insulin and glucagon-like signaling [54].

### 2.2. Genetic Models

Metabolic syndrome negatively affects healthy longevity but takes years to study in mammalian models, thereby delaying the development of translational applications [55]. Therefore, development of genetic mammalian models with shortened lifespan and fast progression to an obese phenotype has become a convenient approach to use for obesity studies.

The leptin-deficient (Lep^ob/ob^), leptin receptor-deficient (LepR^db/db^), and lethal yellow agouti (A^y^/a) mice are the three most commonly used spontaneous mutant obese mouse models. Leptin is a peptide hormone that is secreted by adipocytes and regulates appetite. Leptin and its receptor are key factors in the development of obesity. Leptin resistance is characterized by reduced satiety, overconsumption of nutrients, and increased total body mass [56]. Lep^ob/ob^ mice are homozygous mutants and show obesity, hyperphagia, transient hyperglycemia, glucose intolerance, and elevated plasma insulin [57, 58]. LepR^db/db^ mice manifest morbid obesity, chronic hyperglycemia, and pancreatic beta cell atrophy and become hypoinsulinemic [58–61]. Lep^ob/ob^ and LepR^db/db^ mice are commonly used to model diabetes 2 type and obesity [58, 60, 61]. A^y^/a mice have a mutation at the mouse agouti (a) locus that is associated with an all-yellow coat color, obesity, diabetes, tumors in heterozygotes, and preimplantation embryonic lethality in homozygotes. They display insulin resistance and can even develop diabetes depending on the background strain. Leptin signaling is active in A^y^/a mice that demonstrate a delayed onset in obesity. However, obesity development can be accelerated by using a high-fat diet, making A^y^/a mice a convenient model to study human obesity [62].

MC4R-deficient mice are another very useful strain for use in human obesity research. These mice have a mutation in the melanocortin-4 receptor gene (*Mc4r*), and mutations of the MC4R protein are associated with early-onset obesity in humans. Furthermore, a null *Mc4r* allele in mice leads to severe obesity due to hyperphagia and decreased energy expenditure [63, 64].

Obese Zucker rats (ZDF) are widely used and are among the best genetic rat models for MetS research because these rats display all the conditions of MetS, and several other rat strains were derived from the obese Zucker rats having specific MetS traits [7, 65]. ZDF rats possess a (fa/fa) mutation and are defective in leptin receptor. These animals become obese at the age of 3-5 weeks. At 14 weeks, approximately 40% of their body is already composed of fat. Male ZDF animals develop features of diabetes mellitus. Female rats become obese but do not develop diabetes, maintaining good insulin sensitivity for a prolonged time. ZDF rats develop glucose intolerance, dyslipidemia, hyperphagia, hyperinsulinemia, insulin resistance, endothelial dysfunction, hypertension, proinflammatory, and oxidative status [66].

Short-lived genetically obese DU6 (Titan) mice show increased plasma insulin, leptin, IL-6, and fasting TAG levels. Fat accumulation in pancreas and thymic medullary hyperplasia as well as liver transcriptome and proteome alterations indicates multiple changes in lipid metabolism in Titan mice. Late dietary restriction in these mice demonstrated antiobesity effects including decrease in fat content and improvement of expression of genes involved in lipid synthesis. This supports the use of “Titan” mice as a model of metabolic disorders, systemic inflammation, and early aging [55].

Another mouse model of MetS was developed by crossing aromatase-deficient (ArKO) mice with apolipoprotein E-deficient (ApoE−/−) mice [67]. Double knockout, MetS-Tg mice were generated as a result of successive crossbreeding of ArKO with ApoE−/−-deficient mice. The phenotypic characteristics of the MetS-Tg mice included the increased body weight, central obesity, impaired glucose tolerance, elevated blood pressure and fatty liver, and elevated serum cholesterol and TAG levels as compared with wild-type mice. Thus, this double mutant strain of mice displayed the main clinical features of the MetS [67].

In addition to mammalian models, genetic *Drosophila* models of obesity have also been developed. There are a number of laboratory-generated and naturally occurring genetic variants that make *Drosophila* an ideal model to test the effects of genes on obesity [9]. Genetic screening studies have identified genes that confer obesity in *Drosophila* via TAG quantification. Several conditional *in vivo* gene expression systems, among which the two-component GAL4-UAS system is the most popular, can induce overexpression or RNAi-mediated transgenic gene knockdown in a spatially or temporarily restricted manner. These genetic manipulations allow for analysis of the consequences of obesity without altering diet or the nutrient-sensing pathways [9, 40]. For example, severe obesity can be triggered via inhibition of either lipolytic pathway, one acting via the lipase Brummer and the other via AKH hormone signaling [40, 68–72].

### 2.3. Сhemically Induced Models of MetS

Weight gain is a widely observed side effect of many prescribed drugs, and drug-induced increases in body weight make people more susceptible to obesity-related diseases. Antipsychotics, antidepressants, antihyperglycemics, antihypertensives, and corticosteroids (e.g., dexamethasone) are all medications that are associated with significant weight gain and with a high incidence of MetS [7, 73] that was confirmed in animal studies [7, 74–76]. Literature data suggest that rodents are more suitable models than *Drosophila* for study chemically induced MetS, because many drugs have significant toxic effects on *Drosophila* and flies do not prefer food supplemented with toxicants [77, 78]. Herewith, some chemicals can cause similar metabolic disruptions in both animal groups; in particular, exposure to chemicals frequently used in plastic products such as bisphenol A or phthalates was found to lead to lipid synthesis and triacylglyceride accumulation in mice [79, 80] and *Drosophila* [81, 82].

## 3. Strategies for the Prevention of Metabolic Syndrome

Animal models are widely used not only for investigation of MetS pathogenesis but also for studying the preventive approaches. For humans, four therapies are actively proposed for body weight reduction: calorie restriction (up to a 50% reduction of calories from a normal diet), increased physical activity, behavioral changes, and, in appropriate patients, pharmacologically approved weight-reducing drugs [83, 84]. In general, there is a lot of literature on preventive strategies, covering not only biomedical studies but also psychosocial and public health aspects which are analyzed in detail elsewhere. Here, we only briefly outline how rodent and *Drosophila* models have contributed to our understanding of the preventative approaches.

All mentioned above strategies can be applied to rodent models, whereas *Drosophila* is mostly used to study dietary interventions including dietary restriction and natural-based drugs. Different approaches are developed to modelling dietary restriction: (i) animals have continuous access to food but the amount of food is restricted (caloric restriction), and (ii) intermittent fasting where periods of feeding are alternated with fasting periods [85]. For *Drosophila*, it is easy to manipulate food composition changing both the content and ratio between carbohydrates and proteins in the food. Along with short lifespan, it makes *Drosophila* a very suitable model to study long-term effects of caloric restriction, in particular on lifespan and transgenerational effects. The convenience of applying genomic and metabolic analysis to *Drosophila* allowed to identify key signaling pathways underlying CR effects [86–88]. In rodent models, along with CR, different variants of intermittent fasting, including time-restricted feeding, and every other day fasting are popular approaches that have been proposed for lifespan extension and improvement of health span of elder animals [89–91]. Intermittent fasting is not a common approach to model dietary restriction in *D. melanogaster* possibly due to fast fly metabolism and the doubts about the use of those time frames for food restriction as for mammals and humans. At the same time, there are several studies which report on effectiveness of time-restricted feeding for combating metabolic dysfunction in *Drosophila* model of obesity [92] and restoring cardiac function in aged flies [93].

There is strong evidence that regular exercise contributes to body weight and fat loss and reduces the risk of MetS and obesity. Exercise interventions in humans usually focus on chronic diseases, national fitness, and body weight loss; therefore, it is important to use animal models to investigate the molecular mechanisms underlying the health benefits from regular physical activity. Some reports have shown that endurance exercise can be effective for cardiac function and fat metabolism in *Drosophila* [94, 95] although rodents remain the main models for studying the physiological effects and molecular mechanisms of different exercise programs [96].

Gut microbiota also play an important role in the development of obesity and MetS. MetS is often accompanied by an imbalance of the gut microbiota that leads to a low-grade inflammatory response following by destruction of the gut barrier and development of insulin resistance through metabolites affecting host metabolism and hormone release. Therefore, gut microbiota may be a potential target for the treatment of MetS [97]. Murine models allow manipulations in gut microbiota to be studied in controlled experimental conditions and thus help to assess causal relationship between the host-microbiota interactions and to develop mechanistic hypotheses. In obesity studies, genetically modified models (such as Lep^ob/ob^ leptin-deficient mice) and germ-free mouse models are indispensable because they allow interventions that cannot be performed in humans to provide evidence of how gut bacteria influences host metabolism [98]. In recent years, *D. melanogaster* has become an attractive model for microbiota studies because its gut microbiota has lower diversity, consisting of a small number of species that can be cultivable and easily manipulated [99].

Dietary interventions, including natural-based drugs, are proposed to be an important approach for MetS and obesity management [84, 100]. Various dietary bioactive natural compounds have been shown to be effective in the prevention and treatment of MetS and obesity via targeting of digestion processes, adipocyte proliferation and differentiation, and molecular pathways related to obesity progression and inflammation [100]. Plants rich in phenolic compounds and isolated phenols (catechins, quercetin, curcumin, luteolin, apigenin, resveratrol, etc.) also provide protective effects against MetS and obesity [85, 100, 101], and their antiobesity effects were confirmed in a number of rodent studies [102–104]. Studies on antiobesity agents in *Drosophila* as an alternative model organism of obesity are currently very limited [105] but nutrigenomic approaches in the fruit fly are actively developing that helps to elucidate host-genome interactions with the nutritional environment, including diets and dietary supplements.

When the behavioral and dietary approaches are not sufficient, a pharmacologic treatment is recommended. Pharmacological management of obesity has a long history with multiple disappointments. Numerous drugs were approved for the treatment of obesity; however, most of them were withdrawn because of their adverse effects and insufficient efficacy. The cause of failure has been multifactorial and concerns the limited translational value of animal models to predict cardiovascular safety coupled with considerable patient heterogeneity [106]. Herewith, animals, typically rodents, remain a relevant model to search new therapeutic antiobesity agents. One of the successful pharmacological approaches seems to be using of glucagon-like peptide-1 receptor (GLP1R) to improve metabolism and modest lowering body weight [107]. In obese mice, treatment with semaglutide, a GLP1R agonist, led to consequent weight loss, reduced liver inflammation, insulin resistance, and stress of endoplasmic reticulum [108, 109]. Currently, semaglutide is approved by European Medicines Agency and the Food and Drug Administration for the treatment of type 2 diabetes mellitus and is ongoing clinical trials as antiobesity drug [107]. There is limited information of effectiveness of pharmacological agents in *Drosophila* model of obesity and MetS. It is reported that glibenclamide and rosiglitazone, known antidiabetic drugs showing effectiveness in rodents, have no any effect on the diet-induced metabolic disruption observed in *Drosophila* [110].

## 4. Limitations and Shortcomings of the Animal Models

### 4.1. Rodents

The main rodent models used for the study of obesity and MetS are diet-induced obesity models and genetically modified models, the most common being monogenic animals, that display metabolic disorders as a result of a single mutated gene. Both types of animal models have many advantages for studying MetS and obesity, but there are some limitations that should be taken into account when choosing the most appropriate model.

Monogenic models have the advantage of developing severe metabolic phenotypes that provide more possibilities for therapeutic interventions since the effects of drugs can be faster and better observed. Monogenic models can also save time because pathology progresses more quickly than in diet-induced obesity models [111]. In particular, at 1 month of age, LepR^db/db^ mice are larger/obese when compared to control (heterozygous) littermates, and LepR^db/db^ mice demonstrate higher fat accumulation in the inguinal and axillary regions. In addition, LepR^db/db^ mice also develop frank hyperglycemia by 8 weeks of age [112–114]. To develop obesity and MetS by means of high caloric diet, it usually takes 8-12 weeks but this feeding regimen usually starts when the mouse reaches the age of at least one month; therefore, the total time of the experiment to obtain an obese phenotype is longer than in the case of genetic models. Since the genetic basis is homogeneous and the environmental factors are controlled, the variability in results tends to be smaller, allowing researcher to use fewer animals. At the same time, results obtained from monogenic models may differ from those observed in a heterogenous population, particularly a human one, since obesity is well known to be a multifactorial disease. In addition, with regard to plasma lipid levels and blood pressure, Lep^ob/ob^, LepR^db/db^, and A^y^/a mice fall short of an ideal model for MetS, and researchers should take this into account before choosing them for MetS studies [3]. In this respect, diet-induced obesity models are a better method to develop and disclose molecular mechanisms of human obesity and MetS [115].

Another disadvantage of monogenic animals is the high mortality of certain strains due to ketosis, e.g., db/db mice have a mutation of the leptin receptor and yet are widely used as a model of diabetes type 2. Sophisticated care is also needed for these animals, which can make research more expensive [115]. In general, the cost of a monogenic animal is US$ 100 to US$ 400, varying with the lineage chosen, that may even increase depending on sex, weight, and age chosen for the research. At the same time, Wistar and the Sprague-Dawley rats, that are the most used diet-induced obesity models, can be purchased on average for 20 dollars each [115].

Diet-induced MetS animal models (DIMSM), especially rodent models, are the most commonly used to study the MetS, because of their simplicity and low cost [8]. Rodent DIMSM models develop metabolic abnormalities within a few weeks, as compared with humans that can take years. One of the disadvantages of using these models is that the definition of obesity established for human populations is difficult to apply to animals. In addition, differences in physiology of model animals and humans should be taken into consideration when the results obtained from a DIMSM are interpreted; in particular, in humans, the development of the disease can take years, while in rodents, the observed MetS develops faster, as well as rodents have higher rates of metabolism and differences in immune system that can make the disease symptoms differ between animal species and humans [8].

To get diet-induced MetS animal models, different types of diets are used such as high-carbohydrate diets, high-fat diets, and high-fat high-carbohydrate diets [33, 116, 117]. A recent analysis [8] indicated that high carbohydrate diets сan be recommended for studying the early stages of MetS, before diabetes 2 type onset, whereas high-fat diets and high-fat high-carbohydrate diets induce the severe features of MetS faster. Composition of the diet for control animals is also very important. Differences in the standard chow used can add variability and difficulties in reproducibility of results obtained by different authors [118]. Therefore, researchers should be careful to select a basic or standard food in MetS studies. Standard chow (basic food) is usually made from several agricultural by-products; therefore, the exact content of the various components in the chow remains unknown. High-fat diets are often prepared by adding fats to the basic food. As a result, this leads to a reduction in protein content of the final diet. Lowering protein levels in high caloric diets is undesirable, because low protein intake may lead to a loss of body weight and adipose tissue, which is clearly not the objective of this diet [20, 119]. Therefore, it is recommended that the protein content remains as stable as possible to avoid such alterations. Other disadvantages that can impact the comparison of results from different studies are high variability in the duration of the diet treatment (from 2 to 20 weeks) and variable age of animals at the start of dieting (from 3 to 60 weeks) [8].

### 4.2. Drosophila

A defined cluster of clinical criteria has been established to diagnose human patients and rodent models with MetS. In the case of *D. melanogaster*, not all MetS criteria, especially central obesity and blood pressure, can be applied [120]. For humans, there are already established exact values of clinical parameters for distinguishing healthy persons from sick ones. For *D. melanogaster*, there are no such clear indicators. Researchers are guided only by the parameters of the control group versus the experimental one. However, it is difficult to establish whether the parameters of an experimental fly group are within the normal distribution or beyond the range of healthy parameters. *Drosophila* is a fast and suitable model for screening research on obesity-related genes and certain antiobesity approaches, in particular by measuring levels of storage lipids. However, this model does not allow for a fully assess the pathophysiological consequences of such manipulations proceeding in humans, notably due to the open circulatory system and differences in organ structure and behavior traits.

## 5. Rodents vs. *Drosophila* Models of MetS and Obesity

In terms of structural, physiological, and genetic proximity to humans, rodents seem to be the preferable models for the study of MetS pathophysiology than *Drosophila*. Rodents, especially diet-induced models, can develop all key features of the human MetS [65] whereas *D. melanogaster* does not.

Discovery of leptin, one the main obese genes in mouse [121] inspired further research for identification of the molecular players and pathways involved in adiposity. The studies with gene-targeted mice provided a fundamental contribution to the historical development of understanding the basic parameters that regulate the components of our energy balance [122], and then, these findings have been complemented by studies in lower organisms, including *Drosophila* [68, 123, 124]. Virtually, all key metabolic regulators examined to date display conserved functions across phyla, including, for instance, insulin signaling, mTOR, and key lipases such as ATGL (adipose triglyceride lipase in mammals and its *Drosophila* homolog Brummer lipase) [43, 124, 125]. This level of conservation, together with the power of *Drosophila* genetics, makes the fly a very useful model system to study energy homeostasis and its perturbations [126] in a cost-efficient and fast manner.

Due to easy of genetic manipulations, *Drosophila* show advantages in the study of genetics of obesity as compared with mammals, in particular, in identifying of new genes related to obesity. Taking into account that genetic background of obesity is mostly polygenic, a functional relationship between these candidate genes and adiposity remains a significant challenge in which the fruit fly plays an optimistic role. Genome-wide analysis in *Drosophila* helps to reveal diet-by-gene interactions and uncover diet-responsive genes [127].

Functional screens in cultured cells permit rapid testing of candidate genes, as it was shown in studies of insulin secretion in islet cells for genes associated with type 2 diabetes [128]. However, obesity is a system-level disorder that cannot be replicated in cells. There before, a functional screen *in vivo* is needed, where *Drosophila* is at the forefront [129, 130]. Most studies in *Drosophila* perform forward genetic screens related to obesity before assessing whether misregulation of the corresponding mammalian orthologue affects adiposity [124, 130].

In the study of Pospisilik et al. [124], genome-wide RNAi screening in adult *Drosophila* allowed to identify ∼500 candidate obesity genes. More than 60% of candidate genes identified in that screen were conserved between *Drosophila* and humans, and notably, a large number were previously uncharacterized. In particular, a role for hedgehog signaling was identified as the top-scoring fat-body-specific pathway in *Drosophila* [124] and then confirmed in white/brown adipocyte determination in mice [124, 131]. It links *in vivo* RNAi-based scanning of the *Drosophila* genome to regulation of adipocyte cell fate in mammals [124].

Thus, rodent and *Drosophila* obesity and MetS studies complemented each other and permit to identify conserved and distinct mechanisms underlying metabolic disturbances. Advantages and limitations of different animal obesity models are summarized in Table 2.

## 6. Conclusions

Rats and mice are the most common model of obesity and metabolic syndrome, and *Drosophila* emerges recently as a new model to study metabolic disturbances. Diet, genetic, and chemical-based approaches are developed in both mammalian and insect models to induce obesity and related metabolic disturbances. Whereas genetic models allow fast obtaining disease phenotype, diet-induced obesity models seem to be better to disclose molecular mechanisms and to explore preventive strategies due to obesity is a multifactorial disease. Due to easy genetic manipulations, *Drosophila* seems an attractive model to screening obesity genes. Rodent models have preference in the establishment of pathophysiological complications of MetS. At the same time, the physiological features of both models should be taken into account when extrapolating data to humans.

## Figures and Tables

**Figure 1:** Schematic representation of the approaches used to induce metabolic syndrome in model animals and the consequences of these interventions. The thickness of the arrows means the predominant factor in the induction of key features of MetS.

**Table 1:** Development of MetS traits in selected animal models.

	Elevated blood pressure (hypertension)	Adiposity/obesity	Hyperglycemia/glucose intolerance/insulin resistance	Elevated triglycerides	Reduced HDL/increased total cholesterol
Rodent					
Diet induced (i) HFD-fed C57Bl/6 [16]		**+**	**+**	**+**	**+**
(ii) High fructose diet-fed Wistar rats [34]	**+**	**+**	**+**	**+**	**+**
Monogenic mutants (i) ob/ob mice [58, 61]	**+**	**++**	**+**	**+**	**+**
(ii) db/db mice [58, 61]		**+**	**++**	**+**	**+**
*Drosophila*					
Diet-induced (i) HFD-fed flies [53]		**+**	**+**	**+**	
(ii) High sucrose fed flies [47]		**+**	**+**	**+**	
Monogenic mutants (i) *bmm* mutant [69]		**+**		**+**	
(ii) Mutants in insulin-like peptides (dILPs) [42–44]			**+**	**+**	

**Table 2:** Summary of animal models of MetS and obesity.

Benefits	Limitations
Rodents	
(i) Similarity with humans in anatomy and energy metabolism that allows study pathophysiology of MetS and obesity (ii) Animals reproduce quickly and are relatively easy to handle and transport (iii) Relatively short lifespan; therefore, entire life cycle of animals can be studied within only two or three years (iv) Animals can be inbred to yield genetically identical strains that allowing studying transgenerational effects (v) Relatively easy to study the effects of single genes by developing transgenic animals or gene knockouts to determine the influence of a gene on MetS (vi) High-fat feeding studies require only months to induce MetS	(i) Compared to maintenance of *Drosophila*, rodent husbandry is more expensive (ii) Bioethical limitations; in particular, it restricts using of rodents in screening studies (iii) Some strains do not develop all MetS components or are obesity-resistant, e.g., (1) BALB/c and CBA/J mice are moderate resistant to diet-induced obesity and diabetes (2) Lep^ob/ob^ and LepR^db/db^ mice are resistant to atherosclerotic lesions (3) In many cases, ApoE−/− mice do not become obese, even on HFD (iv) Sexual dimorphism due to diet-induced insulin resistance and glucose intolerance is also observed in rats, with males being the most affected (v) Different high-calorie diets exert different metabolic abnormalities at different times of consumption that affect reproducibility of studies (vi) Many strains (e.g., Lep^ob/ob^ and LepR^db/db^) are susceptible to tumor formation

Drosophila	
(i) Low cost of maintenance in the laboratory (ii) No bioethical limitations (iii) High rate of reproduction and short life cycle allowing fast receiving obese phenotype (~1-2 weeks) and studying transgenerational effects (iv) Short lifespan that allows studying long-term effects of metabolic perturbances (v) Flies contain tissues and organs that are analogous to all those involved in human obesity and associated metabolic diseases (vi) Most genes known to function in metabolic diseases are conserved between flies and humans (vii) *Drosophila* develop obesity and its associated complications during overconsumption of high caloric food, similarly to humans (viii) *Drosophila* insulin induces an increase in fat cell mass, just as in mammals, because insulin acts on triglyceride storage and on fat body cell number (ix) Well-studied genetics and ease of genetic manipulations that allows screening of potential candidates in obesity-associated genes and preliminary screening of antiobesity drugs	(i) Physiological differences: open circulatory system, no veins and arteries, and no blood pressure in hemolymph (ii) Diacylglycerols are the transport form of lipids in *Drosophila* (iii) No abdominal obesity, because a storage fat is accumulated in the fat body, which extends along the dorsal part of the body (iv) Deficiency in insulin-like peptides (dILPs) has different effects on circulating sugar levels, energy storage, and feeding preferences, indicating a divergence in dILP function (v) Due to flight ability, obese phenotype is hard to be developed in population cages

## Data Availability

No data were used to support this study.

## Abbreviations

AKH: Adipokinetic hormone
HFD: High-fat diet
HCHF: High-carbohydrate high-fat diet
TAG: Triacylglycerides
MetS: Metabolic syndrome
LDL: Low density lipoproteins
HDL: High density lipoproteins.
